# The Role of Mesenchymal Stem Cells and Exosomes in Tumor Development and Targeted Antitumor Therapies

**DOI:** 10.1155/2023/7059289

**Published:** 2023-02-14

**Authors:** Enguang Yang, Suoshi Jing, Yuhan Wang, Hanzhang Wang, Ronald Rodriguez, Zhiping Wang

**Affiliations:** ^1^Institute of Urology, Lanzhou University Second Hospital; Key Laboratory of Gansu Province for Urological Diseases; Gansu Nephro-Urological Clinical Center, 730030 Lanzhou, China; ^2^Department of Pathology and Laboratory Medicine, UConn Health, Farmington, CT, USA; ^3^Department of Urology, The University of Texas Health Science Center at San Antonio, 7703 Floyd Curl Drive, San Antonio, Texas 78229-3900, USA

## Abstract

Mesenchymal stem cells (MSCs) can be isolated from various tissues in adults and differentiated into cells of the osteoblasts, adipocytes, chondrocytes, and myocytes. Recruitments of MSCs towards tumors have a crucial contribution to tumor development. However, the role of MSCs in the tumor microenvironment is uncertain. In addition, due to its tropism to the tumor and low immunogenic properties, more and more pieces of evidence indicate that MSCs may be an ideal carrier for antitumor biologics such as cytokines, chemotherapeutic agents, and oncolytic viruses. Here, we review the existing knowledge on the anti- and protumorigenic effect of MSCs and their extracellular vesicles and exosomes, the role of MSCs, and their extracellular vesicles and exosomes as antitumor vectors.

## 1. Introduction

In addition to a large number of immune cells, various other types of stromal cells, including mesenchymal stem cells (MSCs), fibroblasts, endothelial cells, and pericytes, are present in the tumor microenvironment [1]. MSCs could be recruited towards tumors, which have been confirmed in many kinds of tumors [2–10]. Chemokines produced by tumor cells, immune cells, and tumor stromal cells, including CC­chemokine ligand 2 (CCL2), CCL5, CXC­chemokine ligand 12 (CXCL12, also known as SDF1) and CXCL1, are involved in this process [11–14]. Additionally, growth factors such as insulin-like growth factor 1 (IGF1), basic fibroblast growth factor (FGF), vascular endothelial growth factor (VEGF), platelet­derived growth factor (PDGF), and transforming growth factor­*β* (TGF*β*) are found to have a role in the recruitment of MSCs [15–18]. Recruitments of MSCs to tumors have a crucial contribution to tumor fate. The review systematically summarizes the role of mesenchymal stem cells and exosomes in tumor development and targeted antitumor therapies.

## 2. The Antitumorigenic Activity of MSCs

MSCs are considered to be antitumor factors in hematological tumor cell lines, including Jurkat leukemia [19], human erythroid leukemia [20], Burkitt's lymphoma [21], non-Hodgkin's lymphoma [22], and T-cell lymphoma [23], and solid tumor cell lines such as breast cancer [24, 25], hepatocellular carcinoma (HCC) [26, 27], prostate cancer [25, 28], melanoma [29], neck squamous cell carcinoma [30], Kaposi's sarcoma [31], pancreatic tumors [31], and multiple myeloma [32] (showed in Table 1). The mechanism of the antitumor effect of MSCs is multifaceted. Lin et al. showed that the growth of lymphoma cells was inhibited by the molecules secreted by umbilical cord MSCs (UC-MSCs) via the oxidative stress pathway by alteration of antioxidant enzymes [21]. In non-Hodgkin's lymphoma, MSCs induce endothelial cell migration in the Transwell test but promotes endothelial cell apoptosis in direct MSC/endothelial cell cocultures. The cytotoxic activity of MSC requires MSC/endothelial cell contact [22]. The MSCs suppress tumor growth in vivo by inhibiting Akt activity in Kaposi's sarcoma [2]. Type I interferon is expressed in high-density cultured adipose tissue MSCs (AT-MSCs). AT-MSCs and their conditioned medium inhibit the growth of breast cancer MCF-7 cells in vitro [25]. Paracrine factors of human fetal MSCs inhibit liver cancer growth by reducing the activation of IGF-1R/PI3K/Akt signaling [26]. AT-MSCs can effectively inhibit the proliferation and division of HCC cells and induce HCC cell death by downregulating the Akt signaling pathway [27].UC-MSCs inhibit the proliferation of prostate cancer PC-3 cells by activating JNK and downregulating PI3K/AKT signals under coculture conditions [28]. Interactions of bone marrow MSCs (BM-MSCs) with head and neck squamous cell carcinoma cell line PCI-13 decrease the expression of epithelia-mesenchymal transition (EMT) markers via reducing expression of Wnt3, MMP14, and beta-catenin [30]. AT-MSCs induce androgen-responsive and androgen-nonresponsive prostate cancer cell apoptosis via the TGF-*β* signaling pathway [33].

## 3. The Protumorigenic Activity of MSCs

However, studies are arguing for the protumorigenic role of MSCs on tumors, including tumor growth, angiogenesis, metastasis, and resistance to drugs [14]. The mechanism of supporting tumor vasculature of MSCs remains controversial. The biologically active factors secreted by MSCs contribute to the angiogenesis of tumors. Tumor-residing MSCs secreted high levels of VEGF in pancreatic carcinoma, which stimulates angiogenesis and increases microvessel density in the tumor [34]. The secretion of interleukin-6 (IL-6) from MSCs increases the secretion of endothelin-1 (ET-1) in colorectal cancer cells, which activates Akt and ERK in endothelial cells, thus enhancing their capacities for vessel formation [35]. Even more, the differentiation of MSCs into endothelial cells is a direct contribution to blood vessel formation. To examine the differentiation of MSCs into endothelial cells, the MSCs were cultured for several weeks in an endothelial cell culture medium containing VEGF. And the results showed that the expression of typical endothelial cell markers could be detected only in very few MSCs [34]. However, another study showed that melanoma cells educated MSCs to create vascular-like structures in vitro, thereby supporting tumor vasculature [36].

MSCs can facilitate tumor cell migration and invasion, EMT, and the formation of secondary metastatic lesions by a vast array of growth factors, cytokines, and chemokines derived from MSCs. MSC-derived C-C and CXC type chemokines, extracellular matrix modulating factors such as lysyl oxidase, and growth factors such as TGF*β*, FGF, HGF, and EGF critically contribute to metastasis [37].

MSCs can promote tumor resistance to chemotherapy. IL-6, IL-7, IL-8, EGF, and IGF secreted from BM-MSCs induce chemoresistance to paclitaxel in head and neck carcinoma [38]. MSCs activated by platinum-based chemotherapy release two unique fatty acids inducing resistance to multiple types of chemotherapy [39]. Moreover, the clinical benefit of chemotherapy can be enhanced by blocking the release of these fatty acids from MSCs. Timaner et al. thought that MSCs could transform into cancer stem cells (CSCs) to support drug resistance [37].

As described above, some reports claim that MSCs can promote tumor progression, while others report that MSCs have antitumor effects. The observed differences may be due to the inherent biological differences in the source of MSCs, the heterogeneity of MSCs, the interaction of MSCs and their secreted factors with the surrounding microenvironment, and other parameters, such as the dose and time of MSCs administration/analysis, as well as the optimal culture condition [22, 40]. The same amount of human amniotic membrane protein extract has different degrees of antipromoting or mitogenic effects on different tumor cells, indicating that the effect of MSCs may depend on the type of main receptors expressed on specific tumor cells [41]. This is why MSCs derived from different sources and acting in different tumor environments have tumor-promoting or antitumor behaviors.

## 4. MSCs as Antitumor Vectors

More and more evidence indicates that MSCs may be an ideal carrier for antitumor biologics such as cytokines (shown in Table 2), chemotherapeutic agents (shown in Table 3), and oncolytic viruses (shown in Table 4). The main reasons of which are listed as follows: (1) MSCs expressing transgenes maintain long-term expression in the body, because of their low immunogenic properties and the production of immunosuppressive molecules [86]. (2) MSCs show a strong tropism to tumors [2–10]. (3) MSCs have the advantages of less ethical controversy, easy access, and rapid proliferation.

### 4.1. MSCs as Antitumor Vectors of Cytokines

#### 4.1.1. Interleukin (IL)

IL-12 is a heterodimeric proinflammatory cytokine, secreted primarily from antigen-presenting cells. This cytokine has very strong antitumor and antiangiogenic properties [87]. Gene modification of MSCs by infection with an adenoviral or retroviral vector encoding human IL-12 augments the antitumor effect in melanoma, renal cell carcinoma, breast tumor, hepatoma, and glioma [51–57]. The antitumor effects of MSC-IL-12 depend on the stronger tumor-specific T-cell responses [51, 57]. Moreover, the antitumor activity of the MSCs-IL-12 is related to the presence of natural killer (NK) cells and interferon-*γ* (IFN-*γ*) [52]. However, MSCs-IL-12 embedded in Matrigel exhibits significant antitumor effects even in immunodeficient mice lacking T, B, and NK cells, but not in IFN-*γ* knockout mice [51]. Fortunately, the intratumoral expression levels of IL-12 are enhanced by MSCs-IL-12 to be tenfold greater than that of free IL-12 groups in the ultimate stage [55]. A 20-day course of intravenous injection of MSC-IL-12 is without systemic toxic effects [55]. Similarly, the tumor growth is inhibited, and survival is prolonged in ovarian-cancer-bearing mice treated with MSCs-IL-21. The number of IFN-*γ*-secreting splenocytes and NK cytotoxicity significantly increase after MSCs-IL-21 administration [59].

#### 4.1.2. Interferon (IFN)

Type I interferons (IFN-*α* and -*β*) show a variety of antitumor effects, including inhibiting cell proliferation, limiting tumor angiogenesis, inducing cell apoptosis, and activating the host's defense against tumors [88]. Systemic administration of MSCs-IFN-*α* significantly inhibits the growth of B16F10 melanoma cells and prolongs the survival. The result of immunohistochemical analysis reveals the promoted apoptosis and the decreased proliferation and vascular system [42]. IFN-*β* produced by MSCs inhibits the growth of malignant cells such as breast cancer, prostate cancer, bronchioloalveolar carcinoma, lung cancer, tongue squamous cell carcinoma, melanoma, lung metastatic melanoma, and pancreatic tumors metastases to the lung [31, 43–48]. Antitumor effect of IFN-*β* may be related to the increase of apoptosis [45] and NK cell activity [44] and inhibition of Stat3 signaling [43]. However, the combination of MSCs-IFN*β* and anti-inflammatory drugs in the treatment of pancreatic tumors may lose these beneficial effects [31]. INF-*β*-MSCs specifically target tumor cells and do not cause damage to internal organs due to the use of INF-*β* alone [46]. The combination of canine MSCs-IFN-*β* and low-dose cisplatin improves the therapeutic effect of canine melanoma [48]. As a type II interferon, IFN-*γ* is mainly produced by lymphocytes and NK cells and plays an important role in the adaptive cellular immune response against tumors [88]. IFN-*γ* is considered to be a promising antitumor drug; however, the clinical application of the protein form of IFN-*γ* is hindered by serious side effects [89]. IFN-*γ*-modified MSCs selectively induce lung tumor cell apoptosis through the activation of caspase-3 in vitro and inhibit the growth and progression of lung cancer in vivo [50].

### 4.2. Tumour Necrosis Factor-Related Apoptosis-Inducing Ligand (TRAIL)

TRAIL is a member of the tumor necrosis factor (TNF) cytokine superfamily with attractive potent antitumor function owing to its unique competence to target cancerous cells without any harm to adjacent normal cells. This is because the expression of TRAIL-specific receptors, termed death receptors, is significantly higher in cancer cells compared with normal cells [90]. MSCs transduced with a lentiviral vector encoding TRAIL are shown to kill multiple tumor cell lines, including lung cancer, malignant mesothelioma, colon cancer, renal cancer lines, human oral squamous cell carcinoma, and breast cancer [60–62]. MSC full-length TRAIL can induce more powerful cytotoxicity against cancer cells than MSCs soluble form TRAIL and also can defeat cancer cell resistance to recombinant TRAIL [62].

### 4.3. MSCs as Delivery of the Chemotherapeutic Agent

Toxicity and acquired resistance to chemotherapeutic drugs still represent the major obstacles to improving the prognosis of patients with cancer. Improving the targeting delivery of cancer therapies to tumor sites is a key point to decreasing their negative side effects. MSCs have been proposed as cellular vehicles for targeted cancer therapies, thanks to their tumor-homing properties. Taking up and releasing chemotherapeutic drugs is the key to MSC-based therapy. MSCs from different sources, including adipose tissues, bone marrow, dental pulp, interdental papilla, and gingiva, acquire strong antitumor activity after priming with chemotherapeutic drugs such as paclitaxel (PTX), doxorubicin (DOX), gemcitabine (GCB), and pemetrexed (PMX) [63–70]. Salehi et al. [63] monitored the path of PTX transported by dental pulp MSCs and absorbed by breast cancer MCF-7 cells through confocal Raman microscopy. The results showed that PTX could be loaded in the dental pulp MSCs of 100%, while almost 86% of the MCF-7 cells uptake it from the conditioned medium [63]. Brini et al. believed that MSCs from interdental papilla were able to take up and release a sufficient amount of PTX against pancreatic carcinoma in vitro [65]. However, BM-MSCs did not take up and release PMX in effective amounts on mesothelioma, although PTX-loaded BM-MSCs dramatically inhibited mesothelioma proliferation [68]. Therefore, we speculate that MSCs have a certain specificity for the absorption and release of drugs, which may be closely associated with the structure of the drug, the surface protein of the MSCs, and the tolerance of the MSCs to the drug. Considering current research primarily in vitro, whether the MSCs loaded with chemotherapeutic drugs are protected by the immune system in systematic administration remains to be explored.

MSCs or engineered MSCs carried chemotherapeutic drugs may be a promising method for the treatment of drug-resistant tumors. The coculture of ovarian cancer cells with PTX-AT-MSCs inhibited cell viability in 2D and 3D models and counteracted PTX-resistance cells [64]. Coccè et al. demonstrated that AT-MSCs engineered with TRAIL were resistant to PTX and able to incorporate and then release the drug. The PTX delivery together with TRAIL secretion resulted in increased antitumor efficacy in human pancreatic carcinoma and glioblastoma in vitro [66].

The efficiency of drug-loaded nanoparticles is determined by the enhanced permeation and retention effect. As a result, the underperfused or hypoxic location within tumors rarely benefits from nanomedicine [71]. MSCs are recognized as ideal carriers of nanomedicine for tumor-targeting therapy because of their tumor-homing potential in response to proinflammatory cytokines in the tumor microenvironment. MSCs are engineered with drug-loaded nanoparticles and result in an antitumor effect [71–73]. MSCs loaded with nano-PTX result in significant inhibition of tumor growth and superior survival. Furthermore, at doses that result in equivalent therapeutic efficacy, nanoengineered MSCs do not affect white blood cell count, whereas PTX solution and PTX nanoparticle treatments cause leukopenia [72]. A silica nanorattle-DOX drug delivery system is efficiently anchored to MSCs by specific antibody-antigen recognitions at the cytomembrane interface. MSCs-nano-DOX can track down the U251 glioma tumor cells and deliver DOX with wide distribution and long retention lifetime in tumor tissues with low systematic toxicity in vivo [73]. Zhao et al. [71] prepared DOX-loaded poly (d, l-lactic-co-glycolic acid) (PLGA) nanoparticles and loaded them in MSCs. The average DOX content was measured at 20.98 ± 4.02 pg/cell in PLGA-DOX-loaded MSCs, which resulted in improved drug concentration in the lungs and sites of the metastasis and enhanced antitumor efficacy [71].

### 4.4. MSCs as Delivery of Oncolytic Virus

The oncolytic virus (OV) has shown promising results in various clinical trials for the treatment of various cancers. However, systemic administration of OV is severely restricted by their immunogenic nature and poor tumor-homing ability; thus, oncolytic adenovirus (OADV) cannot be utilized to treat disseminated metastases [74]. The MSC-based delivery system which could circumvent humoral immunity is an ideal solution. The success of this strategy depends on efficient ex vivo cellular loading with the virus, intracellular virus amplification, effective cellular targeting of tumor sites following systemic administration, and successful virus hand-off at the tumor site. MSCs acquire strong antitumor activity after transducing with the OVs such as OADV, oncolytic herpes simplex virus (OHSV), and oncolytic measles virus (OMV) (shown in Table 4) [74–85, 91].

It is critical to load viruses into MSCs efficiently ex vivo. Conventional OADV cannot be efficiently loaded into human MSCs due to the low surface expression of coxsackie and adenovirus receptors in MSCs. Na et al. showed that the loading efficiency of OADV into MSCs could be greatly enhanced by complexing the OADV with cationic polymer PCDP, a poly(ethylenimine)- (PEI-) conjugated poly(cystaminebis(acrylamide)-diaminohexane). Furthermore, systemic administration of OADV-PCDP-MSCs elicited a more potent antitumor effect compared to naked OADV alone in the pancreatic tumor model [74].

OVs engineered with molecular methods and then loaded into MSCs can improve virus titers and the effective cellular targeting of tumor sites following systemic administration. Yoon et al. inserted a sequence encoding a Wnt-inhibiting decoy receptor (WNTi) into the OADV that targets alpha-fetoprotein- (AFP-) positive HCCs and then loaded it into MSCs. Both OADV and OADV-MSC elicited minimal killing effects in the normal BJ cell line, showing that the oncolytic effects occur with high specificity toward cancer cells. In the orthotopic HCC tumor model, the systemic administration of OADV-MSC resulted in a markedly 8.1-fold antitumor activity than OADV alone at 35 days postimplantation [75]. OADV deleted the antiapoptotic viral gene E1B19K or downregulated expression of the death ligand TRAIL increased virus titers released from MSCs, which resulted in improved killing of the pancreatic cancer cells [78]. Menstrual blood MSCs (MB-MSCs) combined with ICOVIR15-cBiTE, an OADV expressing an epidermal growth factor receptor- (EGFR-) targeting bispecific T-cell engager (cBiTE), enhanced the antitumor efficacy compared to MB-MSCs loaded with the unarmed virus ICOVIR15 [80]. Guo et al. demonstrated that MB-MSCs specifically targeted tumor cells and served as an OADV delivery platform. MB-MSCs loaded with OADV (CRAd5/F11) inhibited tumor growth in vivo and in vitro [76]. The growth of ovarian cancer lung metastases and breast cancer brain metastases were strongly inhibited after a single injection of MSCs loading OHSV retargeted to HER2 [83]. MSCs-OHSV resulted in significantly increased antiglioblastoma efficacy compared with direct injection of purified OHSV in a preclinical model of glioblastoma resection, ensuing in extended median survival in mice. And MSCs loaded with OHSV-TRAIL successfully induced apoptosis-mediated killing and extended median survival in mice bearing OHSV- and TRAIL-resistant glioblastoma in vitro [81].

Enhancement of antitumor efficacy of MSCs-OV not only benefits from its ability to circumvent humoral immunity to homing but also infiltration of immune cells and differentiation ability of MSCs. MSCs-OMV was protected from antiviral antibodies, which was why therapy with MSCs-OMV resulted in significant inhibition of tumor growth in both measles antibody-naïve and passively immunized SCID mice. By contrast, when OMV was delivered systemically alone, antitumor activity was evident only in measles antibody-naïve SCID mice [84]. Similarly, BM-MSCs enhanced the therapeutic efficacy of systemically delivered OMV in the presence of preexisting high titer anti-MV antibodies in the SCID murine model of acute lymphoblastic leukemia [85]. Rincón et al. suggested that the use of MSCs as carriers of OADV could improve the clinical efficacy of anticancer virotherapy, not only by driving the adenovirus to tumors but also through their potential to recruit T cells, including CD8+ and CD4+ T cells [77]. Intracarotid-delivered MSCs-OHSV, but not purified OHSV, efficiently tracked metastatic tumor deposits in the brain, suppressed brain tumor growth, and prolonged survival in mouse models of melanoma brain metastasis. Furthermore, an increased CD8 + IFN*γ*+ tumor-infiltrating T lymphocytes population was observed after injecting MSC-OHSV intracarotid [82]. Combination therapy of MSCs-OHSV and anti-PD-L1 improved therapeutic efficacy in a syngeneic mouse model of melanoma brain metastasis [82]. The UC-MSC-loaded OADV could be home to the tumor sites and differentiate into hepatocyte-like cells within the tumor microenvironment first. Subsequently, the OADV lysed tumor cells selectively to exhibit tumor inhibition on both orthotopic and subcutaneous hepatic xenograft tumor model mice with less toxicity on normal organs [79].

## 5. Effect of MSC Extracellular Vesicles (EVs)/Exosomes on Tumors

Exosomes derived from MSCs serve as paracrine mediators to inhibit or promote tumor progression by transferring signaling molecules (shown in Table 5). Human UC-MSC-EVs exert potently antiproliferative and proapoptotic results on bladder tumor T24 cells both in vitro and in vivo through restraining phosphorylation of Akt and upregulating p-p53/p21 and cleaved Caspase 3 [92]. EVs derived from human BM-MSCs induce apoptosis to inhibit cell cycle progression and the growth of HepG2 hepatoma, Kaposi's sarcoma, and Skov-3 ovarian tumor cell lines in vitro and in vivo [93]. miR-16 shuttled by MSC-derived exosomes can downregulate the expression of VEGF in tumor cells to suppress angiogenesis and tumor progression in vitro and in vivo [95]. Normal BM-MSC exosomes miR-15a inhibit the growth of multiple myeloma cells, although multiple myeloma BM-MSC-derived exosomes promoted multiple myeloma tumor growth [94]. TRIM14 can promote the proliferation of AML cells via activating PI3K/AKT pathway, which is reversed by BM-MSC exosomes through delivering miR-23b-5p [100].

Nevertheless, it has also been reported that MSC-derived exosomes or EVs are involved in modulating tumor growth and advancing tumor progression. BM-MSC-derived EVs support the tumor growth and angiogenesis of breast cancer in vivo and in vitro [96]. BM-MSC-derived exosomes promote human osteosarcoma and gastric cancer cell proliferation through the activation of the hedgehog signaling pathway [97]. In addition, BM-MSC-derived exosomes enhance VEGF expression in tumor cells by activating the extracellular signal-regulated kinase1/2 (ERK1/2) pathway [98]. AT-MSC-derived exosomes promote migration of the breast cancer cell line MCF7 via activation of the Wnt signaling pathway [99].

It is worth noting that the effects of MSC exosomes or EVs from different sources on the same tumor cell line may be inconsistent. MSC exosomes derived from the same tissue may have different effects on different cell lines. For example, BM-MSC-derived exosomes inhibited the angiogenesis of the murine breast cancer cell line 4T1 [95], while AT-MSC-derived exosomes promote the migration of the human cell line MCF-7 [99]. In addition, BM-MSC-derived EVs promote the proliferation and metastasis of human breast cancer cell line MCF-7 [96]. The effect of protumor or antitumor of MSC exosomes may be related to the source of MSCs, the protocol of MSC culture and exosome extraction, the heterogeneity of cancer cells, and the surrounding microenvironment. Given this, if natural MSC exosomes are used alone to treat tumors, the protocol of MSC culture and exosome extraction must be standardized, and the effects and mechanisms of MSC exosomes for specific tumors must be clarified. In addition, local treatment by intratumoral injection may be safer than systemic administration.

## 6. Extracellular Vesicles and Exosomes Derived from MSCs as Antitumor Vectors

The exosomes are smaller, less complex, and less immunogenic than their parent cells since they have a lower content of membrane-bound proteins [113]. In addition, exosomes contain transmembrane and membrane-anchored proteins that likely enhance endocytosis, thus promoting the delivery of their internal content [114]. As demonstrated by Smyth et al. [115], the internalization of exosomes within tumor cells is ten times greater than liposomes of comparable size, representing a superior specificity of exosomes for cancer targeting. EVs and exosomes derived from MSCs may be ideal antitumor vectors (shown in Table 6).

### 6.1. miRNA

miR-122-transfected AT-MSCs can efficaciously package miR-122 into secreted exosomes, which can mediate the miR-122 conversation between AT-MSCs and HCC cells, thereby rendering cancer cells sensitive to chemotherapeutic agents through alteration of miR-122-target gene expression in HCC cells [106]. Systemic administration of miR-379-enriched EVs causes a significant reduction in tumor activity over the 6 weeks of monitoring [107]. Exosomal miR-9-3p secreted from BM-MSCs inhibits viability, migration, and invasion while promoting apoptosis in bladder cancer via the downregulation of ESM1 [112]. The delivery of miR-139-5p from UC-MSC-derived exosomes results in the repression of proliferation, invasion, and migration of T24 cells together with the inhibition of bladder tumorigenesis in nude mice [101]. BM-MSC-derived exosomes expressing miR-146b inhibit glioma growth via decreasing expression of EGFR and NF-*κ*B protein [104]. BM-MSC-derived exosomes containing miR-143 are easily transferred into recipient cells and suppressed the migration of osteosarcoma cell lines [105]. MSC exosomes are effectively used as a delivery vector to transport PLK-1 siRNA to bladder cancer cells in vitro, resulting in selective gene silencing of PLK-1 [108]. The delivery of anti-miR-9 to the resistant glioblastoma cells reverses the expression of the multidrug transporter and reverses the chemoresistance of glioblastoma cells [103].

### 6.2. Drugs

PTX-loaded MSC-derived EVs are loaded with PTX and possess strong antiproliferative activity on the pancreatic adenocarcinoma cell line CFPAC-1 [102]. PTX-loaded MSC exosomes are successfully isolated using a miniextruder. They significantly decrease the viability of MDA-MB-231 cells of breast cancer in vitro and inhibit tumor growth in vivo [110]. The MSC exosomes loaded with DOX are prepared by mixing exosome with DOX, desalinizing with triethylamine, and then dialyzing against PBS overnight. Compared with the free DOX, the prepared exosome-DOX shows enhanced cellular uptake efficiency and antitumor effect in the osteosarcoma MG63 cell line [111].

## 7. Conclusion and Prospect

Recently, it has been increasingly verified that MSCs play a prominent role in tumor growth, progression, and treatment response. However, the role of MSCs and EVs in tumor progression is controversial, with apparently contradictory results having been published. Such contradicting observations may be related to the heterogeneity of MSCs and experimental condition, such as the dose and time of MSC or EV administration and the optimal culture condition. Generation methods and culture systems of MSCs should be better standardized to make results more reproducible in future research. Furthermore, although MSCs are clinically used as therapeutic agents in inflammatory disease and regenerative medicine, the potential functional role of multipotential differentiation of MSCs during cancer development in vivo is so far uncertain. Large and stringently designed studies are required to answer whether MSCs contribute to carcinogenesis for people without tumors following systemic administration.

Also, because of their tropism to the tumor and low immunogenic properties, MSCs have been recently developed as carriers for against cancer biologics like cytokines, chemotherapeutic agents, and OVs. Few studies focus on the biosafety of engineered MSCs, despite the fact that a small number of MSCs may be present in other regions of the body and may affect healthy tissues after delivery of modified MSCs. As a result, a comprehensive evaluation of the optimal dose, therapeutic routine, drug distribution, and biological safety of engineered MSCs in cancer treatment is required. Furthermore, most of the research examining the efficacy of engineered MSCs on tumors is mainly performed in cancer cells and/or animal models. It would be meaningful to launch clinical studies to demonstrate the safety and efficacy of engineered MSCs in tumors.

Herein, we present several promising research directions for the future. First, MSCs as vehicles of chemotherapeutic drugs augment the targeting delivery of antitumor efficacy to tumor sites and avoid toxicity and acquired resistance to chemotherapy. Next, whether MSC-loaded nanoparticles have an advantage over nanoparticles remains to be seen, such as reduction of nanotoxicity and circumventing immune rejection.

## Figures and Tables

**Table 1:** The antitumorigenic activity and mechanism of MSCs on tumors.

Cancer types	MSC groups	In vivo/in vitro	Phenotypes	Underlying mechanism	References
Kaposi's sarcoma	BM-MSC	In vivo	Inhibit tumor growth	Inhibition of Akt activity	[2]
Jurkat leukemia cells	BM-MSC/UCB-MSC	In vitro	Suppress proliferation; promote apoptosis, differentiation, and drug sensitivity	Unknown	[19]
Erythromyeloblastoid leukaema	UCB-MSC	In vitro	Suppress proliferation	Unknown	[20]
Burkitt's lymphoma cells	UC-MSC	In vitro	Suppress proliferation; promote apoptosis	Via the oxidative stress pathway by alteration of antioxidant enzymes	[21]
Non-Hodgkin's lymphoma	BM-MSC	In vitro and in vivo	Induce endothelial cell migration in the Transwell assay, promote endothelial cell apoptosis in direct MSC/endothelial cell cocultures.	Unknown	[22]
T-cell lymphoma	AT-MSC	In vitro and in vivo	Inhibit tumor growth	Unknown	[23]
Breast cancer	UC-MSC	In vivo and in vitro	Inhibit tumor angiogenesis and increase apoptosis	Unknown	[24]
Breast cancer	AT-MSC	In vitro	Suppress proliferation;	IFN-*β* expressed by MSCs	[25]
Hepatocellular carcinoma	Fetal MSCs	In vivo and in vitro	Suppress proliferation; enhance the therapeutic efficacy of sorafenib and sunitinib	Reduced activation of IGF-1R/PI3K/Akt signaling	[26]
Hepatocellular carcinoma	AT-MSC	In vitro	Suppress proliferation;	Downregulation of Akt signaling	[27]
Prostate cancer	UC-MSC	In vivo and in vitro	Suppress proliferation; induce apoptosis	Activation of JNK and downregulation of PI3K/AKT signaling	[28]
Melanoma	AT-MSC	In vivo and in vitro	Suppress proliferation; induce apoptosis	Unknown	[29]
Neck squamous cell carcinoma	BM-MSC	In vitro	Suppress the onset of EMT	Reduced expression of Wnt3, MMP14, and beta-catenin	[30]
Pancreatic tumors	BM-MSC	In vivo	Inhibit tumor growth	Unknown	[31]
Multiple myeloma	UC-MSC	In vitro and in vivo	Inhibit tumor growth and tumor progression	Unknown	[32]
Prostate cancer	AT-MSC	In vitro and in vivo	Suppress proliferation; induce apoptosis	TGF-*β* signaling pathway	[33]

MSC: mesenchymal stem cells; UC-MSC: umbilical cord MSC; AT-MSC: adipose tissue MSC; BM-MSC: bone marrow MSC; EMT: epithelial-mesenchymal transition; UCB-MSCs: umbilical cord blood-derived mesenchymal stem cells.

**Table 2:** MSCs as antitumor vectors of cytokines.

Cancer types	MSC groups	In vivo/in vitro	Agents	Methods	Routes of administration	Main results	References
Melanoma lung metastasis	BM-MSC	In vivo	IFN-*α*	Adenoviral vectors	i.v.	Reduce the growth of lung metastasis in melanoma and prolonged the survival	[42]
Melanoma and breast cancer	BM-MSC	In vivo and in vitro	IFN-*β*	Adenoviral vectors	Coculture in vitro and i.v. in vivo	Inhibit tumor cell growth and suppress the growth of pulmonary metastases	[8]
Pancreatic tumor	BM-MSC	In vivo	IFN-*β*	Adenoviral vectors	i.p.	Suppress tumor growth	[31]
Breast cancer	MSC	In vivo and in vitro	IFN-*β*	Lentiviral gene transfer plasmid	i.v.	Suppress breast cancer growth and reduce pulmonary and hepatic metastases	[43]
Prostate cancer lung metastasis	BM-MSC	In vivo	IFN-*β*	Adeno-associated virus	i.v.	Reduce pulmonary metastases	[44]
Bronchioloalveolar carcinoma	UC-MSCs	In vitro and in vivo	IFN-*β*	Adenoviral vectors	i.v.	Inhibit growth and progression by increasing apoptosis.	[45]
Lung cancer	UC-MSCs	In vivo	IFN-*β*	Lentiviral vectors	i.v.	Delay tumor growth	[46]
Tongue squamous cell carcinoma	G-MSC	In vitro and in vivo	IFN-*β*	Lentiviral vectors	i.v.	Inhibit the proliferation	[47]
Melanoma	Canine AT-MSCs	In vitro and in vivo	IFN-*β*	Lentiviral vectors	i.p.	The combination of MSC-IFN-*β* with low-dose cisplatin improves therapeutic efficacy against canine melanoma.	[48]
Melanoma	BM-MSC	In vivo and in vitro	IFN-*β*	Adenoviral vectors	Coculture in vitro and i.v. in vivo	Inhibited the growth of malignant cells in vivo	[49]
Lung carcinoma	BM-MSC	In vitro and in vivo	IFN-*γ*	Lentiviral vectors	Coculture in vitro and s.c. in vivo.	Induced apoptosis in vitro Inhibited the growth and progression in vivo	[50]
Melanoma	BM-MSC	In vivo	IL-12	Adenoviral vectors	i.t.	Exhibited stronger tumor-specific T-cell responses and antitumor effects	[51]
Renal cell carcinoma	BM-MSC	In vivo	IL-12	Adenoviral vectors	i.v.	Reduced the growth of 786-0 RCC and significantly prolonged mouse survival	[52]
Breast cancer	BM-MSC	In vivo	IL-12	Retroviral vectors	s.c.	Antiangiogenesis and interfere with the growth of 4T1 breast cancer	[53]
Glioma	UCB-MSCs	In vivo	IL-12	Adenoviral vectors	i.t.	Inhibited tumor growth and prolonged the survival of glioma-bearing mice	[54]
Melanoma, breast tumor, and hepatoma	BM-MSC	In vivo	IL-12	Adenoviral vectors	i.v.	Induction of the tumor cell elimination in B16 melanoma, 4T1 breast tumor, and HCA hepatoma cancer	[55]
Malignant glioma	BM-MSC	In vivo and in vitro	IL-2	Adenoviral vectors	i.t.	Inhibition of 9 L tumor growth and increased the survival	[56]
Melanoma	BM-MSC	In vivo	IL-2	Retroviral plasmids	s.c.	Development of CD8-mediated tumor-specific immunity and delay of tumor growth	[57]
Ovarian cancer	AF-MSCs	In vivo	IL-2		i.v.	Migrate to the ovarian cancer tumor site to secrete the functional IL-2 and treat the tumor	[58]
Ovarian cancer	UCB-MSCs	In vivo	IL-21	Transfected with the recombinant pIRES2-IL-21	i.v.	Inhibit tumor growth and prolong the survival	[59]
Malignant mesothelioma	BM-MSC	In vivo/in vitro	TRAIL	Lentiviral vectors	Coculture in vitro i.v. in vivo	Kill multiple malignant mesothelioma cell lines in vitro and reduce mesothelioma tumor growth in vivo	[60]
Lung cancer	BM-MSC	In vitro	TRAIL	Lentiviral vectors	In vitro coculture	Reduce the growth of primary cancers and metastases	[61]
Various cancer cell lines	BM-MSC	In vitro	TRAIL	Lentiviral vectors	In vitro coculture	Defeat cancer cell resistance to recombinant TRAIL	[62]

MSC: mesenchymal stem cells; UC-MSC: umbilical cord MSC; AT-MSC: adipose tissue MSC; BM-MSC: bone marrow MSC; UCB-MSCs: umbilical cord blood-derived mesenchymal stem cells; IL: interleukin; TRAIL: tumor necrosis factor-related apoptosis-inducing ligand; G-MSC: gingiva-derived mesenchymal stromal cells; IFN: interferon.

**Table 3:** MSC as delivery of chemotherapeutic agent.

Cancer type	MSC group	In vivo/in vitro	Agents	Methods	Main results	Reference
Breast cancer	Dental pulp MSCs/BM-MSCs	In vitro	PTX	Incubated for 12 h with 10 *μ*M PTX	Induce apoptosis	[63]
Ovarian cancer	AT-MSC	In vitro	PTX	Exposed to 2 *μ*g/mL PTX for 24 h	Inhibit ovarian cancer spheroid growth and overcome paclitaxel resistance	[64]
Pancreatic carcinoma	Interdental papilla MSCs	In vitro	PTX	Exposed to 2 *μ*g/mL PTX for 24 h	Against pancreatic carcinoma cells	[65]
Pancreatic carcinoma and glioblastoma	AT-MSCs	In vitro	PTX	MSCs were engineered with TRAIL	MSCs-TRAIL primed with PTX resulted in an increased antitumor efficacy	[66]
Oral squamous cell carcinoma	G-MSC	In vitro	PTX, DOX, GCB	Exposed to 2 *μ*g/mL PTX, DXR, or GCB for 24 hours	Inhibition of squamous cell carcinoma growth	[67]
Malignant pleural mesothelioma	BM-MSC	In vitro	PTX, PMX	Exposed to 2 *μ*g/mL PMX or PTX for 24 h	Inhibit the in vitro proliferation	[68]
Breast cancer, anaplastic thyroid cancer	BM-MSC	In vivo and in vitro	DOX	Incubated for 12 h with 5 *μ*M DOX	Enhanced cytotoxic effects	[69]
Pancreatic cancer	BM-MSC/MSC derived from pancreatic tissues	In vitro	GCB	Subconfluent MSC cultures (3–4 × 10^5^ cells) were exposed to 2000 ng/mL of GCB. Twenty-four hours later	Inhibit the growth	[70]
Lung melanoma metastases	AT-MSC	In vivo and in vitro	Nano-DOX	PLGA-DOX with the concentration ranging from 10 *μ*g/mL to 100 *μ*g/mL were incubated with 1 × 10^5^ MSCs for 1 h	Improved drug concentration in the lungs and sites of metastasis and enhanced antitumor efficacy	[71]
Lung carcinoma	BM-MSC	In vivo	Nano PTX	Incubated with nano-PTX (100 *μ*g/mL) for 4 h at 37°C with occasional stirring	Significantly improved anticancer efficacy at a considerably reduced dose of the drug	[72]
Glioma	BM-MSC	In vivo and in vitro	Nano -DOX	A final concentration of 100 *μ*g/mL or 1 mg/mL nano-DOX was added to the cells and incubated for different times	Increased and prolonged intratumoral drug distribution results in enhanced tumor cell apoptosis.	[73]

MSC: mesenchymal stem cells; UC-MSC: umbilical cord MSC; AT-MSC: adipose tissue MSC; BM-MSC: bone marrow MSC; UCB-MSCs: umbilical cord blood-derived mesenchymal stem cells; G-MSC: gingiva-derived mesenchymal stromal cells; PTX: paclitaxel; DOX: doxorubicin; GCB: gemcitabine; PMX: pemetrexed.

**Table 4:** MSC as delivery of oncolytic virus.

Cancer types	MSC groups	In vivo/in vitro	Agents	Route of administration	Main results	Reference
Pancreatic tumor	BM-MSCs	In vivo and in vitro	OADV	i.v.	Tumor growth inhibition by induction of apoptotic cell death and degradation of tumor extracellular matrix	[74]
Hepatocellular carcinoma	BM-MSCs	In vivo and in vitro	OADV	i.v.	OADV-MSC resulted in markedly 8.1-fold antitumor activity than OADV alone at 35 days postimplantation	[75]
Colorectal cancer	MB-MSCs	In vivo and in vitro	OADV(CRAd5/F11)	Coculture in vitro i.v. in vivo	Inhibit tumor growth	[76]
Lung cancer	AT-MSCs	In vivo an in vivo	OADV(ICOVIR5)	i.t.	Inhibit the growth of tumors in vivo	[77]
Pancreatic cancer	BM-MSCs	In vitro	OADV		Improved tumor cell killing	[78]
Hepatocellular carcinoma	UC-MSCs	In vivo and in vitro	OADV	i.v.	Tumor inhibition on both orthotopic and subcutaneous hepatic xenograft tumor model mice	[79]
Lung adenocarcinoma	MB-MSCs	In vivo	OADV(ICOVIR15-cBiTE)	i.p.	ICOVIR15-cBITE-loaded MB-MSCs enhance antitumor efficacy	[80]
Malignant glioblastoma	BM-MSCs	In vivo and in vitro	OHSV	Stereotactically implanted into the brains	Induce apoptosis-mediated killing and prolonged median survival	[81]
Brain metastatic melanomas	MSC and mMSC	In vivo and in vitro	OHSV	Intracarotid	Track metastatic tumor deposits in the brain, suppress brain tumor growth and prolong survival in mouse models of melanoma brain metastasis	[82]
Breast cancer metastases to the brain/ovarian cancer lung metastases	Fetal membrane-derived MSCs	In vivo	OHSV	i.v.	Tumor growth inhibition of lung and brain metastases	[83]
Liver cancer	BM-MSCs	In vivo	OMV	i.v.	Inhibition of tumor growth in both measles antibody-naïve and passively-immunized SCID mice	[84]
Acute lymphoblastic leukemia	BM-MSCs	In vivo	OMV	i.v.	Inhibition of cancer development in a murine model of disseminated ALL following MSC-mediated delivery of OMV	[85]

MSC: mesenchymal stem cells; UC-MSC: umbilical cord MSC; AT-MSC: adipose tissue MSC; BM-MSC: bone marrow MSC; OV: oncolytic virus; OADV: oncolytic adenovirus; OHSV: oncolytic herpes simplex virus; OMV: oncolytic measles virus.

**Table 5:** Effect of MSC extracellular vesicles EVs/exosomes on tumors.

Cancer type	Source of MSC	In vivo/in vitro	Agents	Mechanism	Interacting cells	Results	References
Bladder cancer	UC-MSC-derived MVs	In vivo and in vitro	Unknown	Downregulated phosphorylation of Akt protein kinase and upregulated cleaved caspase 3	T24	Antiproliferation and proapoptosis	[92]
Hepatoma/Kaposi's sarcoma/ovarian tumor	BM MSC-derived MVs	In vitro and in vivo	Unknown		HepG2 hepatoma, Kaposi's sarcoma, and Skov-3 ovarian tumor cell lines	Induced apoptosis and inhibit the growth	[93]
Multiple myeloma	Exosomes derived from normal BM MSCs	In vitro and in vivo	Unknown	miR-15a in exosomes derived from normal BM MSCs	Multiple myeloma cells	Inhibited the growth	[94]
Breast cancer	BM-MSC-derived exosomes	In vitro and in vivo	miR-16	miR-16 suttled by MSC-derived exosomes reduces the VEGF expression	Mouse breast cancer cell line (4T1)	Suppress angiogenesis	[95]
Breast cancer	BM MSCs EVs	In vitro and in vivo	miR-21 and miR-34a		MCF-7	Supported breast cancer cell proliferation and metastasis possibly by transferring miR-21 and miR-34a	[96]
Osteosarcoma and human gastric cancer	BM MSC exosomes	In vitro	Unknown	Activation of hedgehog signaling pathway	Osteosarcoma (MG63) and gastric cancer (SGC7901) cells	Promoted tumor growth.	[97]
Gastric cancer	BM-MSC-derived exosomes	In vivo	Unknown	Enhanced VEGF expression in tumor cells by activating the ERK1/2 pathway	SGC-7901 cells	MSC-exosomes promote tumor angiogenesis and cell proliferation in vivo	[98]
Breast cancer	AT-MSC-derived exosomes	In vitro	Unknown	Activation of the Wnt signaling pathway	MCF7	Promote migration	[99]
Acute myeloid leukemia	BM-MSC-derived exosomes	In vitro	miR-23b-5p	Inhibit the function and expression of TRIM14	THP-1	Induced the apoptosis	[100]

MSC: mesenchymal stem cells; UC-MSC: umbilical cord MSC; AT-MSC: adipose tissue MSC; BM-MSC: bone marrow MSC; EVs: extracellular vesicles; MVs: microvesicles.

**Table 6:** Extracellular vesicles and exosomes derived from MSCs as antitumor vectors.

Cancer types	MSC groups	In vivo/in vitro	Agents	Methods	Mechanisms	Results	References
Bladder cancer	UC-MSC-derived exosomes	In vivo/in vitro	miR-139-5p	UCMSCs transfected with miR-139-5p mimic or miR-139-5p inhibitor	Downregulate the PRC1 expression	Suppressed proliferation, migration, and invasion potentials	[101]
Pancreatic adenocarcinoma	BM-MSC-derived MVs	In vitro	PTX	MSCs were exposed to 2 *μ*g/mL PTX for 24 h		Suppressed proliferation	[102]
Temozolomide-resistant glioblastoma	BM-MSC-derived exosomes	In vitro	miR-9 inhibitor			Reverse the chemoresistance	[103]
Glioma	BM-MSC-derived exosomes	In vivo	miR-146b	Cel-miR-67 and hsa-miR-146b expression plasmids were used for electroporation of MSC.	Decreasing EGFR and NF-*κ*B protein	Inhibit glioma growth	[104]
Osteosarcoma	BM-MSC-derived exosomes	In vitro	miR-143	Transfection		Reduced the migration of osteosarcoma cells	[105]
Hepatocellular carcinoma	AT-MSC-derived exosomes	In vivo/in vitro	miR-122	Transfected with plasmids of hsa-miR-122 or cel-miR-67	Downregulation of CCNG1, IGF1R, and ADAM10	Increase chemosensitivity	[106]
Breast cancer	BM-MSC-derived EVs	In vivo/in vitro	miR-379	Lentiviral transduction	Downregulation of COX-2	Reduced tumor activity over the 6 weeks of monitoring	[107]
Bladder cancer	MSC-derived exosomes	In vitro	siRNA of PLK-1	Electroporation	Knockdown of PLK-1 mRNA	Transfer PLK-1 siRNA to bladder cancer cells	[108]
Glioma	BM-MSCs, AT-MSCs, UC-MSC-derived EVs	In vitro and in vivo	miR-124/miR-145 mimics	Transfected with the miR mimics by electroporation, lentiviral transduction	Downregulates the expression of SCP-1	Reduced the tumor cells migration and the stem cell properties of glioma cells	[109]
Breast cancer	BM-MSC-derived exosomes	In vitro and in vivo	PTX	Extrusion with varying pore sizes (10, 5, and 1 *μ*m) in a miniextruder (Avanti Polar Lipids)		Decreased the viability and inhibited tumor growth	[110]
Osteosarcoma	BM-MSC-derived exosomes	In vitro	DOX	The 70 *μ*L of Dox HCl (1 mg mL^−1^) was mixed with 930 *μ*L exosome solution (1 mg mL^−1^) for 30 min and desalinized with triethylamine for 1 hr at room temperature (RT)		Suppressed proliferation	[111]
Bladder cancer	BM-MSC-derived EVs	In vivo and in vitro	miR-9-3p		miR-9-3p targets ESM1	Inhibits viability, migration, and invasion while promoting apoptosis	[112]

MSC: mesenchymal stem cells; UC-MSC: umbilical cord MSC; AT-MSC: adipose tissue MSC; BM-MSC: bone marrow MSC; EVs: extracellular vesicles; MVs: microvesicles; PTX: paclitaxel; DOX: doxorubicin.

## Abbreviations

MSCs: Mesenchymal stem cells
IGF1: Insulin-like growth factor 1
VEGF: Vascular endothelial growth factor
PDGF: Platelet­derived growth factor
TGF*β*: Transforming growth factor­*β*
UC-MSC: Umbilical cord MSC
AT-MSC: Adipose tissue MSC
HCC: Hepatocellular carcinoma cells
BM-MSC: Bone marrow MSC
EMT: Epithelia-mesenchymal transition
IL: Interleukin
NK: Natural killer cells
TRAIL: Tumour necrosis factor-related apoptosis-inducing ligand
TNF: Tumor necrosis factor
PTX: Paclitaxel
DOX: Doxorubicin
GCB: Gemcitabine
PMX: Pemetrexed
OV: Oncolytic virus
OADV: Oncolytic adenovirus
OHSV: Oncolytic herpes simplex virus
OMV: Oncolytic measles virus
AFP: Alpha-fetoprotein
EGFR: Epidermal growth factor receptor
EVs: Extracellular vesicles
AF-MSCs: Human amniotic fluid mesenchymal stem cells
UCB-MSCs: Human umbilical cord blood-derived mesenchymal stem cells
G-MSC: Gingiva-derived mesenchymal stromal cells
IFN: Interferon
MB-MSCs: Menstrual blood-derived mesenchymal stem cells
CSCs: Cancer stem cells
MVs: Microvesicles.
